The article "Gastroprotective effect of desmosdumotin C isolated from Mitrella kentii against ethanol-induced gastric mucosal hemorrhage in rats: possible involvement of glutathione, heat-shock protein-70, sulfhydryl compounds, nitric oxide, and anti-Helicobacter pylori activity" was retracted in 2024. Reasons: duplicated images; overlap with earlier publications; unreliable results or conclusions; concerns about the authorship.

# Gastroprotective effect of desmosdumotin C isolated from *Mitrella kentii* against ethanol-induced gastric mucosal hemorrhage in rats: possible involvement of glutathione, heat-shock protein-70, sulfhydryl compounds, nitric oxide, and anti-*Helicobacter pylori* activity

**DOI:** 10.1186/1472-6882-13-183

**Published:** 2013-07-19

**Authors:** Heyam Mohamed Ali Sidahmed, Ainnul Hamidah Syahadah Azizan, Syam Mohan, Mahmood Ameen Abdulla, Siddig Ibrahim Abdelwahab, Manal Mohamed Elhassan Taha, A Hamid A Hadi, Kamal Aziz Ketuly, Najihah Mohd Hashim, Mun Fai Loke, Jamuna Vadivelu

**Affiliations:** 1 Department of Pharmacy, Faculty of Medicine, University of Malaya, Kuala Lumpur 50603, Malaysia; 2 Department of Molecular Medicine, Faculty of Medicine, University of Malaya, Kuala Lumpur 50603, Malaysia; 3 Department of Chemistry, Faculty of Science, University of Malaya, Kuala Lumpur 50603, Malaysia; 4 Medical Research Centre, Jazan University, P.O. Box 114, Jazan, Saudi Arabia; 5 Department of Medical Microbiology, Faculty of Medicine, University of Malaya, Kuala Lumpur 50603, Malaysia

## Abstract

**Background:**

*Mitrella kentii* (*M. kentii*) (Bl.) Miq, is a tree-climbing liana that belongs to the family Annonaceae. The plant is rich with isoquinoline alkaloids, terpenylated dihydrochalcones and benzoic acids and has been reported to possess anti-inflammatory activity. The purpose of this study is to assess the gastroprotective effects of desmosdumotin C (DES), a new isolated bioactive compound from *M. kentii*, on gastric ulcer models in rats.

**Methods:**

DES was isolated from the bark of *M. kentii*. Experimental rats were orally pretreated with 5, 10 and 20 mg/kg of the isolated compound and were subsequently subjected to absolute ethanol-induced acute gastric ulcer. Gross evaluation, mucus content, gastric acidity and histological gastric lesions were assessed *in vivo*. The effects of DES on the anti-oxidant system, non-protein sulfhydryl (NP-SH) content, nitric oxide (NO)level, cyclooxygenase-2 (COX-2) enzyme activity, bcl-2-associated X (Bax) protein expression and *Helicabacter pylori* (*H pylori*) were also investigated.

**Results:**

DES pre-treatment at the administered doses significantly attenuated ethanol-induced gastric ulcer; this was observed by decreased gastric ulcer area, reduced or absence of edema and leucocytes infiltration compared to the ulcer control group. It was found that DES maintained glutathione (GSH) level, decreased malondialdehyde (MDA) level, increased NP-SH content and NO level and inhibited COX-2 activity. The compound up regulated heat shock protein-70 (HSP-70) and down regulated Bax protein expression in the ulcerated tissue. DES showed interesting anti-*H pylori* effects. The efficacy of DES was accomplished safely without any signs of toxicity.

The article "Gastroprotective effect of desmosdumotin C isolated from Mitrella kentii against ethanol-induced gastric mucosal hemorrhage in rats: possible involvement of glutathione, heat-shock protein-70, sulfhydryl compounds, nitric oxide, and anti-Helicobacter pylori activity" was retracted in 2024. Reasons: duplicated images; overlap with earlier publications; unreliable results or conclusions; concerns about the authorship.

**Conclusions:**

The current study reveals that DES demonstrated gastroprotective effects which could be attributed to its antioxidant effect, activation of HSP-70 protein, intervention with COX-2 inflammatory pathway and potent anti *H pylori* effect.

## Background

Gastric ulcer is a common disease affecting many people worldwide [1]. Some factors that are identified in the etiology of this disorder include stress, cigarette smoking, alcohol consumption, nutritional deficiencies and infections [2]. However, the over-ingestion of non-steroidal anti-inflammatory drugs (NSAIDs) and *H pylori* infection remains the predominant cause of peptic ulcer disease [3]. The gastric ulcer disease was observed to correlate with changes in several physiological parameters, such as Reactive oxygen species (ROS), NO, lipid peroxidation and gastric acid over secretion [4]. Treatment of gastric ulcer is considered a clinical problem due to the increasingly widespread use of NSAIDs and low-dose aspirin [5]. Despite the effectiveness of reciprocal antiulcer drugs such as the antacids, anticholinergics, proton pump inhibitors and histamine H-2 receptor antagonists, the majority of them possess adverse effects that limit their usage [6]. Nowadays, the pursuit to discover alternative therapies to treat gastric ulcer is of high concern [7]. A large number of natural antiulcer compounds have been isolated from medicinal plants and the common chemical classes of bioactive compounds that have been identified as possessing antiulcer activity are the alkaloids, saponins, xanthones, triterpenes and tannins, among others [8].

*M. kentii* is a tree-climbing liana which belongs to the family Annonaceae. The plant is native to Peninsular Malaysia, several parts of Indonesia including the islands of Sumatra and Borneo as well as New Guinea. In Malaysia, *M. kentii* is used traditionally as a drink in the form of a root decoction to treat fever [9]. Experimentally, the plant showed anti-inflammatory activity [10]. Previous chemical studies on *M. kentii* resulted in the isolation of isoquinoline alkaloids [11], terpenylated dihydrochalcones [12] and four other benzoic acids [10]. As a continuation of our research for biologically active compounds for the treatment of gastric ulcer from the Malaysian flora, a hexane extract of the bark of this plant was selected for phytochemical investigations. For the first time, our study led to the isolation of DES (Figure 1) from *M. kenti*. It is a known compound which was previously isolated from the roots of *Desmos dumosus*[13] and *Uvaria schefferi*[14].

The article "Gastroprotective effect of desmosdumotin C isolated from Mitrella kentii against ethanol-induced gastric mucosal hemorrhage in rats: possible involvement of glutathione, heat-shock protein-70, sulfhydryl compounds, nitric oxide, and anti-Helicobacter pylori activity" was retracted in 2024. Reasons: duplicated images; overlap with earlier publications; unreliable results or conclusions; concerns about the authorship.

**Figure 1:** Chemical structure of desmosdumotin C.

It is known that ethanol induces gastric mucosa lesions and petechial bleeding in humans [15], where ethanol is found to penetrate easily and rapidly into the gastric mucosa and causes membrane damage, exfoliation of cells, erosion and ulcer formation. It is claimed that ROS are involved in the ulcer formation caused by ethanol [16]. Ethanol-induced gastric ulcer models are commonly used to study both the pathogenesis of and therapy for human ulcerative diseases [2].

DES has a unique chalcone skeleton, and it is known that naturally occurring chalcones have shown interesting bioactivities such as antimalarial, antitumor, anti-HIV and anti-oxidant effects [17]. However, the compound has not been well-studied so far to evaluate its bioactivites, except for its significant and selective in vitro cytotoxicity toward cancer cell lines [13]. Based on these prospective activities of its chemical structure, the current study is conducted to evaluate for the first time the gastroprotective effect of DES from *M. kentii* and possible mechanism(s) involved against ethanol-induced ulcer model in rats.

## Methods

### Plant materials

The bark of *M. kentii* was collected in Mersing, Johor. A voucher specimen (KL 4139) is deposited at the Herbarium of Department of Chemistry, University of Malaya, Kuala Lumpur, Malaysia.

### Extraction and isolation of DES

The dried and powdered bark (1.0 kg) of *M. kentii* was extracted exhaustively with hexane using Soxhlet extractor. The hexane extract was concentrated under reduced pressure to give a residue. Hexane crude extract was subjected to column chromatography (CC). The isolation and purification of DES were carried out by chromatography on a small column silica gel (0.040-0.063 mm) using n-hexane: ethyl acetate, 9:1 as a solvent system. DES, C_19_H_20_O_4_, was isolated as a yellow needle crystal from a n-hexane – CH_2_Cl_2_ mixture, m.p.: 93–94 °C; UV ( _methanol_ : 380, 242, 225 nm; IR_max_ (cm^-1^, NaCl disc) : 3401, 1657, 1624, 1577, 1513, 1426, 1371, 1243, 1153, 1122, 977, 944; EIC-MS m/z [M + H]^+^ (%) : 312.140729 (calc. 312.3646 for C_19_H_20_O_4_); ^1^H NMR (CDCl_3_, TMS) ( (ppm): 8.32 (1H, d, J = 16Hz), 7.92 (1H, d, J = 16Hz), 7.66 (2H, m, Ar-2”,6”-H), 7.37 (3H, s, Ar-3”, 4”, 5”-H), 3.93 (3H, s, OCH_3_), 2.02 (3H, s, Ar-CH_3_) 1.36 (6H, s, CH_3_ × 2). ^13^C NMR (CDCl_3_, TMS) ( (ppm) : 198.14 (C-1), 192.48 (C-3), 187.26 (C-1’), 176.70 (C-5), 144.94 (C-2’, 3’), 135.29 (C-1”), 130.66 (C-3”, C-5”), 128.98 (C-4”), 123.30 (C-2”, 6”), 113.68 (C-2), 106.67 (C-4), 62.23 (OCH_3_), 50.49 (C-6), 24.44 (CH_3_ × 2), 9.88 (Ar-CH_3_). The compound was identified by comparison of their spectroscopic data with literature values.

The article "Gastroprotective effect of desmosdumotin C isolated from Mitrella kentii against ethanol-induced gastric mucosal hemorrhage in rats: possible involvement of glutathione, heat-shock protein-70, sulfhydryl compounds, nitric oxide, and anti-Helicobacter pylori activity" was retracted in 2024. Reasons: duplicated images; overlap with earlier publications; unreliable results or conclusions; concerns about the authorship.

### Chemicals and drugs

TPTZ, DTNB, Griess reagent were purchased from Sigma-Aldrich Chemical Co. Kuala Lumpur, Malaysia. Indomethacin and omeprazole were obtained from University of Malaya Medical Center. All other used chemicals and reagents were of analytical grade.

### Animals

Healthy ICR mice (6–8 weeks old weighing 20–30 g) and Sprague Dawley rats (200–220 g) were obtained from the Experimental Animal House, Faculty of Medicine, University of Malaya. All procedures relating to animal care and the animal research protocols conformed to the animal care guidelines of the Institutional Animal Care and Use Committee, University of Malaya. This study specifically was presented to the institutional ethical review board (UM ICUCA) for approval, and the approval was granted [Ethic No FAR/29/06/2012/HMAS (R)]. The animals were fed standard pellets and free access to water ad libitum. All animals received human care according to the criteria outlined in the “Guide for the Care and use of Laboratory Animals “prepared by the National Academy of Sciences and published by the National Institute of Health.

### Acute toxicity study

Thirty six mice (18 male, 18 female) were assigned equally into three groups. Overnight fasted animals received DES at doses of 30 and 300 mg/kg body weight according to Organization for Economic Co-operation and Development (OECD) Guideline 420 protocol year 1992. Animals treated with 5% Tween 80 were served as a control group. The food was withheld for further 3–4 h after dosing. During14 days of treatment, the animals were observed for any mortality or physiological changes. On day 15, body weight variation was determined and all the animals anesthetized using ketamine and xylazil to collect Serum for biochemical analysis then sacrificed. the liver and kidney were excised for histology study.

### Induction of acute gastric lesion

To avoid coprophagy, each rat was kept in a cage with a raised floor of wide mesh and all animals divided randomly into six groups (n = 6). The animals were fasted overnight prior for oral pre-treatment (5 ml/kg b.w) as mention in Table 1.

**Table 1:** animal group with different pretreatment

**Animal group**	**Pretreatment**
Group (A) normal control	Rats pretreated with vehicle (5% Tween 80 v/v) + vehicle) (5% Tween 80 v/v).
Group (B) ulcer control	Rats pretreated with vehicle (5% Tween 80 v/v) + absolute ethanol).
Group (C) reference control	Rats pretreated with 20 mg/kg of omeprazole in vehicle + absolute ethanol).
Group (D)	Rats pretreated with 5 mg/kg of DES in vehicle + absolute ethanol).
Group (E)	Rats pretreated with 10 mg/kg of DES in vehicle + absolute ethanol).
Group (F)	Rats pretreated with 20 mg/kg of DES in vehicle + absolute ethanol).

The pre-treatments were administered for 1 hour, subsequently; all groups except the normal group (A) received absolute ethanol (5 ml/kg). 1 h later, the animals anesthetized using ketamine & xylazil and their blood was collected from their jugular veins for serum biochemical analysis. The animals were then sacrificed and their stomachs were removed immediately [18].

The article "Gastroprotective effect of desmosdumotin C isolated from Mitrella kentii against ethanol-induced gastric mucosal hemorrhage in rats: possible involvement of glutathione, heat-shock protein-70, sulfhydryl compounds, nitric oxide, and anti-Helicobacter pylori activity" was retracted in 2024. Reasons: duplicated images; overlap with earlier publications; unreliable results or conclusions; concerns about the authorship.

### Gastroprotective assessments

Each stomach of the experimental animals was opened along the greater curvature and the stomachs were washed with ice normal saline. Gastric ulcer on the gastric mucosa appears as elongated bands of hemorrhagic lesions. The length (mm) and width (mm) of each band was measured using planimeter [(10 mm × 10 mm = ulcer area) under dissecting microscope (1.8×)]. The area of each ulcer lesion was measured by counting the number of small squares, 2 mm × 2 mm, covering the length and width of each hemorrhagic band. The sum of the areas of all lesions for each stomach was applied in the calculation of the ulcer area (UA) wherein the sum of small squares × 4 × 1.8 = UA mm^2^. The inhibition percentage (I%) was calculated by the following formula described in [19] with slight modifications:

$$\begin{array}{l} \text{The inhibition percentage}\left(I\%\right)\\ \;=\left[\left(\mathrm{UAcontrol}–\mathrm{UAtreated}\right)/\mathrm{UAcontrol}\right]\times 100\% \end{array}$$

### Gastric tolerability test

Each experimental stomach was observed under an illuminated magnifier (3×) to evaluate the gastric lesions according to the modified scoring system of [20] (0:no lesions; 0.5: slight hyperaemia or ≤ 5 petechiae; 1: ≤ 5 erosions ≤ 5 mm in length; 1.5: ≤ 5 erosions ≤ 5 mm in length and many petechiae; 2: 6–10 erosions ≤ 5 mm in length; 2.5: 1–5 erosions > 5 mm in length; 3: 5–10 erosions >5 mm in length; 3.5: >10 erosions >5 mm in length; 4: 1–3 erosions ≤ 5 mm in length and 0.5-1 mm in width; 4.5: 4–5 erosions ≤ 5 mm in length and 0.5-1 mm in width; 5: 1–3 erosions > 5 mm in length and 0.5-1 mm in width; 6: 4 or 5 grade 5 lesions; 7: ≥6 grade 5 lesions; 8: complete lesion of the mucosa with hemorrhage).

### Determination of gastric secretion

The effect of DES on gastric acid output was determined following the recommended method [21]. Briefly, Sprague Dawley rats assigned equally into five groups (n = 6). After 24 h fasting, immediately after pylorus ligature, 5% Tween 80, omeprazole (30 mg/kg), and DES (5, 10 and 20 mg/kg) were administered intraduodenally. 4 hours later, all animals sacrificed by cervical dislocation, their stomachs were removed immediately and the gastric content was collected to determined gastric secretion volume (ml), pH value using digital pH meter and total acidity by titrating with 0.01 N sodium hydroxide using phenolphthalein as indicator and was expressed as mEq/l.

The article "Gastroprotective effect of desmosdumotin C isolated from Mitrella kentii against ethanol-induced gastric mucosal hemorrhage in rats: possible involvement of glutathione, heat-shock protein-70, sulfhydryl compounds, nitric oxide, and anti-Helicobacter pylori activity" was retracted in 2024. Reasons: duplicated images; overlap with earlier publications; unreliable results or conclusions; concerns about the authorship.

### Measurement of mucus content

The gastric mucosa of each animal was gently rubbed off using a glass slide and the weight of the collected mucus was measured using precise electronic balance [22].

### Serum biochemical assays

Serum samples were analyzed at University of Malaya Medical Centre using Hitachi Auto-analyzer to evaluate changes in serum biochemical parameters.

### Histological evaluation

A small fragment of the gastric wall from each animal was fixed in 10% buffered formalin solution followed by tissue dehydrated with alcohol and xylene. Then, each sample was embedded in paraffin wax, sectioned at 5 μm in slides prior for staining. Hematoxylin and eosin (H & E) stain was used for light microscopy [23]. Moreover, to evaluate mucus production, some slides were also stained by periodic acid Schiff Base (PAS) following the manufacture instruction (Sigma Periodic Acid-Schiff (PAS) Kit). For further analysis, other slides underwent for immunohistochemistry (IHC) staining using Dako ARK™ to observed immunhistochemical localization of HSP-70 (1:100) and Bax (1:50) proteins. Both proteins were purchased from Santa Cruz Biotechnology, Inc., California, USA.

### Preparation of gastric tissue homogenate

A specimen of gastric wall from each animal was homogenized (10%) in ice cold 0.1 mol/l phosphate buffered saline (PBS). The homogenates were centrifuged at 10,000 g for 15 min at 4°C. The pure supernatant was used to quantify the gastric tissue contents of GSH, MDA, NP-SH and NO.

### GSH levels

Total GSH content (nmol GSH/g tissue) was estimated by interaction with DTNB (5,5 -dithiobis-2-nitrobenzoic acid) and the absorbance was read in a spectrophotometer (412 nm) [24] .

### Thiobarbituric acid reactive substance assay

Thiobarbituric acid reactive substance (TBARS) assay was used to estimate MDA content. According to [25], the gastric homogenate was added to a 0.126 ml solution containing 26 mM thiobarbituric acid, 0.26 M HCL, 15% trichloroacetic acid and 0.02% butaylated hydroxyltoluene. The mixture was incubated in a water bath at 95°C for 1 h. After cooling, the mixture was centrifuged at 3000 g for 10 min. The absorbance was read in a spectrophotometer at 532 nm and the results were expressed in μmol/g tissue MDA. Tetramthoxy propane was used as standard.

### Estimation of NP-SH content

Gastric mucosal NP-SH (μmol/g of tissue) were measured according to the method of [26]. Briefly, aliquots of 5 ml of the gastric homogenates were mixed with a solution containing 4 ml of distilled water and 1 ml of 50% trichloroacetic acid. The mixture was vortex for 15 min and centrifuged at 3000 × g. 2 ml of supernatant was mixed with 4 ml of 0.4 M Tris Buffer at pH 8.9; 0.1 ml of DTNB [5,5 dithiobis-(2-nitrobenzoic acid)] was added and the sample was shaken. The Absorbance was recorded within 5 min of the addition of DTNB at 412 nm against a reagent blank with no homogenate.

The article "Gastroprotective effect of desmosdumotin C isolated from Mitrella kentii against ethanol-induced gastric mucosal hemorrhage in rats: possible involvement of glutathione, heat-shock protein-70, sulfhydryl compounds, nitric oxide, and anti-Helicobacter pylori activity" was retracted in 2024. Reasons: duplicated images; overlap with earlier publications; unreliable results or conclusions; concerns about the authorship.

### NO level

NO content was quantified by measuring nitrite/nitrate concentration using Griess assay [27]. In brief, gastric homogenates were deproteinated with absolute ethanol for 48 h at 4°C, then centrifuged at 12000 g for 15 min at 4°C. To an aliquot of the supernatant, vanadium trichloride 0.8% (w/v) in 1 M HCl was added for the reduction of nitrate to nitrite, followed by the rapid addition of Griess reagent (sigma) and the absorbance at 540 nm was measured. The results were expressed as (μmol/g tissue). Sodium nitrite was used as standard.

### *In vitro* evaluation of COX-2 inhibitory activity

The COX-2 inhibitory activity of DES was estimated using a COX-inhibitor screening Kit (Cayman Chemical, USA). According to the manufacturer’s instructions, DES was dissolved in DMSO at final concentration was 0–100 μg/ml. The inhibition was calculated by the comparison of compound treated to control incubations. Indomethacin was used as reference standard.

### Ferric-reducing antioxidant power (FRAP) assay

The FRAP value of DES was estimated according to the method of [28] with slight modification. Briefly, the FRAP reagent was prepared freshly from acetate buffer (pH 3.6), 10 mM TPTZ [ 2,4,6-Tri(2-pyridyl)-s-triazine] solution in 40 mM HCl and 20 mM iron (III) chloride solution in proportions of 10:1:1 (v/v), respectively. 50 μl of the compound were added to 1.5 ml of the FRAP reagent in the dark, 4 min later the absorbance was then recorded at 593 nm. The standard curve was constructed linear (R2 = 0.9723) using iron (II) sulfate solution (100–1000 μM), and the results were expressed as μM Fe (II)/g dry weight of the compound.

### DPPH assay method

The scavenging activity of the DES was evaluated according to the recommended method of [29]. Briefly, the compound was mixed with 0.3 mM DPPH [2,2-diphenyl-1-picrylhydrazyl] /ethanol solution to give final concentrations of the compound (50, 25, 12.5, 6.25 μg/ml in ethanol. 30 min later, the absorbance was observed at 518 nm then converted into a percentage of antioxidant activity expressed as the inhibition concentration at 50% (IC50).

### *In vitro* anti-*H pylori* activity

*H pylori* strain, J99 (ATCC 700824) was cultured with brain heart infusion broth (BHI; Oxoid) supplemented with 10% horse serum (Invitrogen) incubated at 37°C in a humidified CO_2_ incubator (Forma Steri-Cycle) for 3 days. Minimum inhibitory concentration (MIC) was determined by a modified microtiter broth dilution method on sterile 96-well polypropylene microtitre plates with round-bottom wells (Eppendorf). Briefly, DES was dissolved and diluted in 5% DMSO to give a 10× working stock solution. *H. pylori* was diluted to a final concentration of 2 × 106 CFU/ml in culture medium. Aliquots of 10 μl of DES were added to 90 μl of *H. pylori* in a well of the microtitre plate. Concentration of DES ranged from 31.25 to 250 μg/ml. The microtiter plate was incubated for 3 days in a CO_2_ incubator. The plate was examined visually and measured using a microplate reader (Varioskan Flash) at 600 nm to determine the lowest concentration showing complete growth inhibition, which was recorded as the MIC. Wells containing *H. pylori* with 10 μl of 5% DMSO and BHI medium containing 250 μg/ml DES, were used as control and blanks respectively. The result was recorded in accordance with the Clinical and Laboratory Standards Institute [30].

The article "Gastroprotective effect of desmosdumotin C isolated from Mitrella kentii against ethanol-induced gastric mucosal hemorrhage in rats: possible involvement of glutathione, heat-shock protein-70, sulfhydryl compounds, nitric oxide, and anti-Helicobacter pylori activity" was retracted in 2024. Reasons: duplicated images; overlap with earlier publications; unreliable results or conclusions; concerns about the authorship.

### Statistical analysis

All tests were performed at least in triplicates and the values were represented as mean ± S.E.M (standard error mean). The statistical differences between groups were determined according to SPSS version 16.0 and Graph Pad prism 6 using ordinary one-way ANOVA followed by Dunnetts multiple comparison tests. A value of P < 0.05 was considered significant.

## Results

### Toxicity study

The toxicity study showed no toxic symptoms or mortality and there were no abnormal physiological or behavioral changes, body weight alteration at any time of observation up to 300 mg/kg during the experimental period. Histological examination to the liver and kidney and the serum biochemical analysis didn’t show any differences incomparable to the control group (data not shown but available upon request).

### Gross evaluation

Pre-treatment with DES at doses of 5, 10, 20 mg/kg b.w and omeprazole at 20 mg/kg significantly (p < 0.05) reduced the ulcer area formation by 69.77%, 90.18%, 86.56% and 79.07%, respectively, compared to the ulcer control. Table 2 shows the statistical significant differences between treatment groups subjected to ethanol induced gastric ulcer. Macroscopic observation showed that DES pre-treated groups (Figure 2D, 2E and 2F) or omeprazole group (Figure 2C) considerably reduced gastric lesion compared to the ulcer control group; where ethanol induced intense gastric mucosal damage in the form of elongated band of hemorrhages (Figure 2B).

The article "Gastroprotective effect of desmosdumotin C isolated from Mitrella kentii against ethanol-induced gastric mucosal hemorrhage in rats: possible involvement of glutathione, heat-shock protein-70, sulfhydryl compounds, nitric oxide, and anti-Helicobacter pylori activity" was retracted in 2024. Reasons: duplicated images; overlap with earlier publications; unreliable results or conclusions; concerns about the authorship.

**Table 2:** Gastroprotective effect of desmosdumotin C against ethanol-induced ulceration and observed liver function test

**Animal group**	**Pre-treatment 5 ml/kg**	**Mucus weight**	**Ulcer area**	**Inhibition (%)**	**ALT**	**AST**
					**(IU/L)**	**(IU/L)**
A	Normal control	2.9 ± 0.2 *	0.00	0.00	36.57 ± 1.67*	230 ± 9.81 *
B	ulcer control	0.98 ± 0.3	557.28 ± 6.2	NA	56.5 ± 2.71	293 ± 2.15
C	Omeprazole (20 mg/kg)	1.55 ± 0.2*	108 ± 7.7 *	79.07	48.2 ± 2.5 *	275.7 ± 6.01 *
D	DES (5 mg/kg)	1.37 ± 0.5 *	168.48 ± 9 * $	69.77	51 ± 1.47 *	283.6 ± 4.39 *
E	DES (10 mg/kg)	2.09 ± 0.1 *#$	54.72 ± 3.8* $	90.18	32 ± 2.8 *#$	240.04 ± 3.79 *$#
F	DES (20 mg/kg)	1.5 ± 0.4 *	74.88 ± 10.3 *$	86.56	34.2 ± 1.6 *$	257.4 ± 9.22*$

*NA*, not applicable; *AST*, Aspartate transaminase; *ALT*, Alanine Aminotranferase. All values are represented as mean (n = 3–5 animals) ± standard error mean, * indicates (p < 0.05) compared to ulcer control. $ indicates (p < 0.05) statistical differences compared to omeprazole group.

**Figure 2:** **Gross evaluation.** Macroscopic appearance of the gastric mucosa of the rats pre-treated with DES at doses 5, 10, 20 mg/kg **(D**,**E**, **F)** or omeprazole 20 mg/kg **(C)** showed reduced lesion formation when compared to the ulcer control rats **(B)** 2C. Ethanol-induced sever injuries to the gastric mucosa appear as elongated bands of haemorrhage (white arrow). **(A)** Showed normal macroscopic appearance of the intact stomach from normal group. (magnification: 1.8×).

### Gastric tolerability

DES animal groups didn’t exhibit any significant gastric lesions. The changes observed in the range of 0–1 according to Adami scoring scale. Only few petechiae scored in rat stomach regardless of a given dose.

### Gastric acidity

In animal model using ligated pylorus method, the treatment with DES (5, 10 and 20 mg/kg) and omeprazole (30 mg/kg), respectively, reduced the volume of gastric juice, total acidity and raised gastric pH significantly (p < 0.05) compared to the control group (Table 3).

**Table 3:** Effects of DES and omeprazole, administered intraduodenally, on the biochemical parameters of gastric juice obtained from pylorus-ligature in rats

**Animal group**	**treatment 5 ml/kg**	**Volume (ml)**	**pH**	**Acid output [H**^**+**^**] mEq/L**
A	Control group (5% Tween 80)	3.5 ± 0.015	3.83 ± 0.088	95 ± 0.88
B	Omeprazole (30 mg/kg)	2.71 ± 0.015^*^	6.17 ± 0.015^*^	83 ± 1.15^*^
C	DES (5 mg/kg)	3.1 ± 0.12^* $^	4.92 ± 0.012^*$^	92 ± 0.58^*$^
D	DES (10 mg/kg)	2.87 ± 0.12^*^	5.98 ± 0.01^*^	89 ± 0.88^*$^
E	DES (20 mg/kg)	2.94 ± 0.008^*^	5.96 ± 0.01^*$^	90 ± 0.33^*$^

Results are expressed as mean ± S.E.M. (n = 6 rats).* indicate p < 0.05 compared to control group. $ indicate p < 0.05 compared to omeprazole.

The article "Gastroprotective effect of desmosdumotin C isolated from Mitrella kentii against ethanol-induced gastric mucosal hemorrhage in rats: possible involvement of glutathione, heat-shock protein-70, sulfhydryl compounds, nitric oxide, and anti-Helicobacter pylori activity" was retracted in 2024. Reasons: duplicated images; overlap with earlier publications; unreliable results or conclusions; concerns about the authorship.

### Gastric mucus content

The ulcer control group produced the lowest content of gastric mucus, while the pretreated DES groups or omeprazole group significantly (p < 0.05) increased the mucus production compared to the ulcer control group (Table 2).

### Serum biochemical analysis

Serum analysis showed that the rats in ulcer control had increased levels of the liver enzymes; Aspartate transaminase (AST) and Alanine Aminotranferase (ALT). However, in DES pretreated animals, the serum concentration of this biomarker significantly (p < 0.05) lowered than ulcer control (Table 2).

### Histological evaluation

Histological observation using H&E staining further confirm the ability of DES to prevent ethanol-induce gastric damage in the superficial layer of the gastric mucosa compared to the normal control group (Figure 3A). The ulcer control group showed highly extensive gastric lesion, submucosal edema and leucocytes infiltration (Figure 3B). Pre-treatment with DES (Figure 3D, 3E and 3F) and omeprazole (Figure 3C), have relatively better protection as observed by decreasing ulcer area, reduced or complete absence of edema and leucocytes infiltration and flattening of mucosal fold was also observed.

**Figure 3:** **Histological evaluation.** The gastric mucosa of the rats pretreated with DES at doses 5, 10, 20 mg/kg **(D**, **E**, **F)** or omeprazole **(C)** showed improved histological appearance compared to ulcer control rats **(B)** which have extensive visible hemorrhagic necrosis of the gastric mucosa with edema and leucocytes infiltration of submucosa. The black arrow indicates edema in submucosa and the white arrow indicates disruption to the deep mucosa layer. **(A)** showed normal histological apperance of the intact stomach from normal group. (H & E stain: 20×).

### Mucus staining

PAS staining was used to observe the glycogen level in control and pretreated animals. DES pre-treatment (Figure 4D, 4E and 4F) or omeprazole (Figure 4C) resulted into the expansion of a substantially continuous PAS-positive mucous gel layer that lining the entire gastric mucosal surface observed as a magenta color. However, gastric specimen from ulcer control group didn’t exhibit this magenta staining color of PAS (Figure 4B).

**Figure 4:** **Tissue glycoprotein.** Effect of DES on gastric tissue glycoprotein-PAS staining in ethanol-induced gastric ulcer in rats where **(A)** normal group, **(B)** ulcer group, **(C)** omeprazole group, **(D**, **E**, **F)** treated DES groups at doses 5, 10 and 20 mg/kg, respectively, where the black arrows indicates the glycoprotein appear as magenta stain (PAS stain 20×).

The article "Gastroprotective effect of desmosdumotin C isolated from Mitrella kentii against ethanol-induced gastric mucosal hemorrhage in rats: possible involvement of glutathione, heat-shock protein-70, sulfhydryl compounds, nitric oxide, and anti-Helicobacter pylori activity" was retracted in 2024. Reasons: duplicated images; overlap with earlier publications; unreliable results or conclusions; concerns about the authorship.

### HSP-70 and Bax immunohistochemistry

Using immunhistochemistry staining, the immunostained localization of HSP-70 was up regulated in DES pretreated animals more than that observed in ulcer control group (Figure 5). This result indicates the possible participation of this protein in protective effect of DES. On the other hand, the immunostained localization of the pro-apoptotic Bax protein in all experimental animals was down regulated compared to the ulcer control group (Figure 6). Hence, the suppressive effect on Bax protein in treatment group might be contributed in the gastroprotective activity of DES. The antigen site in immunohistochemistry appears as a brown-colored.

**Figure 5:** **Immunohistochemical analysis of Hsp-70 protein.** HSP-70 expression in the gastric tissue of rats submitted to ethanol-induced gastric mucosal lesions at different groups where **(A)** normal control group, **(B)** ulcer control group **(B)**, **(C)** omeprazole group, **(D**, **E**, **F)** the pre-treated groups with DES at doses 5, 10 and 20 mg/kg, respectively. The antigen site appears as a brown color (IHC: 20×).

**Figure 6:** **Immunohistochemical analysis of Bax protein.** Bax expression in the gastric tissue of rats submitted to ethanol-induced gastric mucosal lesions at different groups where **(A)** normal control group, **(B)** ulcer control group, **(C)** omeprazole group, **(D**, **E**, **F)** pre-treated group with DES at doses 5, 10 and 20 mg/kg, respectively. The antigen site appears as a brown color (IHC: 20×).

### Effect of DES on GSH and MDA level

GSH as endogenous antioxidant, its level was significantly (p < 0.05) lowered in ulcer control group than the other groups. DES in the pre-treated animals was significantly (p < 0.05) restored the GSH levels that depleted due to ethanol administration (Figure 7A). MDA was used as indicator for lipid peroxidation. Thus, TBARS assay showed that the ulcer control group significantly (p < 0.05) has higher MDA level into the gastric homogenate than the other pretreated groups. Gastric MDA level significantly (p < 0.05) decreased in DES pretreated group’s (Figure 7B).

**Figure 7:** **Effect of DES on gastric tissue homogenate content of (A) Glutathione (GSH), (B) Malondialdehyde (MDA), (C) Non protein sulfhydryl (NP-SH) and (D) Nitric oxide (NO).** DES pre-treatment significantly increased GSH, decreased MDA and replenished NP-SH and NO content. Statistical analysis was assessed with ordinary one way ANOVA followed by Dunnett ’ s Multiple comparison tests. All values are represented as mean of 3 – 5 animals. ± SEM. * indicates (p < 0.05) compared to ulcer control. $ indicates (p < 0.05) statistical differences compared to omeprazole group.

The article "Gastroprotective effect of desmosdumotin C isolated from Mitrella kentii against ethanol-induced gastric mucosal hemorrhage in rats: possible involvement of glutathione, heat-shock protein-70, sulfhydryl compounds, nitric oxide, and anti-Helicobacter pylori activity" was retracted in 2024. Reasons: duplicated images; overlap with earlier publications; unreliable results or conclusions; concerns about the authorship.

### Effect of DES on NP-SH compounds content

The ulcer control group showed the lowered NP-SH level into the gastric homogenate, while DES significantly (p < 0.05) elevated NP-SH level in pretreated animal compared to ulcer control group (Figure 7C).

### Effect of DES on NO level and COX-2 enzyme

Ulcer control showed the lowest level of NO. DES pre-treatment significantly (p < 0.05) has increased NO level into the gastric homogenate compared to ulcer control group. However, none of the treatment was able to increase NO level near to the normal control (Figure 7D). Moreover, DES inhibited COX-2 enzyme activity by 29.5% and 34.8% at 250 and 500 ng/ml, respectively compared with standard COX-2 inhibitor, indomethacin (71.37%) (Figure 8).

**Figure 8:** **Inhibition of COX-2 enzyme.** DES was observed to inhibit COX-2 catalyzed prostaglandin biosynthesis by 29.5% and 34.8% at 250 and 500 ng/ml, respectively, compared with indomethacin as COX-2 inhibitor shows inhibition of 71.37%. The results represent as mean ± SEM.

### Antioxidant evaluation of DES

FRAP and DPPH assays were used to evaluate DES radical scavenging activity. FRAP assay showed that DES has antioxidant capacity with 120.7 ± 2.40 which is significantly (p < 0.05) lowered than the positive control used in this study those exhibiting 2562.7 ± 56.64 and 879.3 ± 10.00, for Gallic acid and Ascorbic acid, respectively (Figure 9). Meanwhile the DPPH assay showed insignificant inhibition in the dose of DES used in this study (data not shown). Therefore, it could be said that the antioxidant effect of DES is probably through indirect antioxidant mechanism.

**Figure 9:** **Ferric reducing/antioxidant power assay.** The FRAP value (μM Fe (II)/g dry mass) of DES in compare with that of ascorbic acid and gallic acid.

### *In vitro* anti-*Hpylori* activity

DES represents interesting MIC with 125 μg/ml against *H. pylori* J99.

## Discussion

In this study, the gastroprotective activity of DES was evaluated on ethanol-induced ulcer model in rats. The effects of DES on the antioxidant system and COX-2 enzyme activity, as well as its anti *H. pylori* effect were also assessed. The ethanol model is widely used to evaluate gastroprotective activity, since ethanol is found to penetrate easily and rapidly into the gastric mucosa, causing membrane damage, exfoliation of cells and erosion. This subsequently increases mucosal permeability together with the release of vasoactive products, which result in gastric lesions and gastric ulcer formation [31]. Ethanol-induced gastric ulcer predominantly affects the glandular portion of the stomach. However, in the present study, DES pre-treatment was found to significantly attenuate ethanol induced-gastric ulcer. The purpose of the following discussion is to evaluate the possible mechanisms that underlie the observed gastroprotective effect of DES.

The article "Gastroprotective effect of desmosdumotin C isolated from Mitrella kentii against ethanol-induced gastric mucosal hemorrhage in rats: possible involvement of glutathione, heat-shock protein-70, sulfhydryl compounds, nitric oxide, and anti-Helicobacter pylori activity" was retracted in 2024. Reasons: duplicated images; overlap with earlier publications; unreliable results or conclusions; concerns about the authorship.

In order to define the side effects of DES on the overall physiological function, serum biochemical parameters were evaluated. In our study, when compared to the normal group, animals in the ulcer group showed an increased serum level of the liver enzymes (AST and ALT) as an indicator of hepatic injury, since a high level of hepatic enzymes is a sign of alcoholic tissue damage due to ethanol administration [32]. However, DES pre-treatment showed a significant decrease in the elevated serum level of the liver enzymes, close to the normal control level. This finding indicates the high efficacy of the compound against ethanol-induced tissue injuries.

Reactive oxygen species (ROS) are the final products generated from a normal cellular metabolic process [33]. Oxidative stress results from the accumulation of ROS and the inability of the antioxidant system to overcome them. Thus, in this situation, excessive production of ROS affects cell integrity [34] such as in gastric tissue where oxidative stress was reported earlier to contribute in the gastrointestinal mucosal lesion formation [35]. Antioxidants have been observed to protect gastric mucosa from ulceration [33], where antioxidants are compounds that have the ability to protect against tissue damage through radical scavenging mechanism [36]. A previous study proved that ethanol induced gastric tissue injury by increasing reactive species formation [37]. Subsequently, ROS accumulation depleted GSH level and increased lipid peroxidation [34]. GSH is an intracellular antioxidant that inhibits oxidative stress [38] and plays an important protective role against ethanol-induced gastric cell injury [39]. It was observed that the aggressive effect of ethanol on gastric mucosa is associated with reduced GSH level [40]. Apart from GSH, ethanol exerts its allergenic effect on gastric tissue by increasing lipid peroxidation [41] where MDA is the main product of lipid peroxidation. Therefore, MDA is considered a marker of ROS-mediated gastric lesions [42]. The present study shows that pre-treatment with DES significantly protected the gastric mucosa from ethanol-induced ulceration by restoring the depleted GSH level and reducing the elevated MDA level compared to the ulcer control group. These results showed the ability of DES to reduce oxidative stress. Hence, to further evaluate this antioxidant property, FRAP assay was used and the results indicated that the compound possesses weak radical scavenging activity. Meanwhile, there is insignificant inhibition in the DPPH assay. Therefore, it could be suggested that DES inhibited oxidative stress via the cellular antioxidant mechanism.

The article "Gastroprotective effect of desmosdumotin C isolated from Mitrella kentii against ethanol-induced gastric mucosal hemorrhage in rats: possible involvement of glutathione, heat-shock protein-70, sulfhydryl compounds, nitric oxide, and anti-Helicobacter pylori activity" was retracted in 2024. Reasons: duplicated images; overlap with earlier publications; unreliable results or conclusions; concerns about the authorship.

Heat shock proteins (HSPs) are stress proteins that maintain the cellular homeostasis against stress factors [43]. HSP70 over expression occur in response to various stimuli such as heat, drug exposure or oxidative stress [44]. Acute and chronic gastric ulcers in rats were observed to be associated with HSP70 induction [43]. HSP70 expression enhances cellular protection-tolerances against high concentration of alcohol [45]. Experimentally, it was found that there is a correlation between HSP induction and mucosal protection [46]. Many compounds have been reported to protect the tissue from oxidative damage remarkably through their activities as HSPs inducers [47]. Our study observed that DES pre-treatment followed by ethanol administration resulted in HSP70 over expression in experimental gastric tissue, suggesting that induction of HSP70 might contribute to the protective effect of DES against ethanol-induced gastric injuries. Again, this result supports the hypothesis regarding the antioxidant activity of DES against oxidative stress.

It was reported earlier that apoptosis or programmed cell death was believed to be one of the main factors that contributes in gastric ulcer formation. Blocking of apoptotic cell death is among the mechanisms that are implicated to control gastric lesions [48]. Apart from the antisecretory effect of omeprazole, it was recently proved to exert its antiulcer action via anti-apoptotic effect [49]. Ethanol was reported to induce gastric mucosal lesion by increasing apoptotic cell death [37]. In many experimental ulcer models, apoptosis results from the alteration of Bcl-2 anti-apoptotic and Bax pro-apoptotic proteins expression [48]. Bcl-2 Proteins inhibit most types of apoptotic cell death [50], while Bax proteins boost this process [48]. In the results presented herein, IHC assay showed that DES was able to suppress Bax protein expression when compared to the ulcer control group. Hence, as DES exerted Bax protein suppression effect, it might be suggested that anti-apoptotic effect is involved in the gastroprotective activity of DES against ethanol-induced gastric tissue injury.

Gastric defensive mechanisms are based mainly on the delicate balance between aggressive and protective factors [51]. Several studies suggest that mucus gel layer is the first defensive mechanism of the mucosa against internal and external aggressive factors [52]. Ethanol tends to disrupt the gastric mucosal layer and lowers the level of tissue proteins [53]. Hence, the compound that has the ability to increase mucus production might be expected to possess gastroprotective activity [54]. To evaluate this effect, DES was subjected to PAS staining and the result revealed the capability of DES to maintain gastric mucus integrity against depletion by ethanol administration. NP-SH plays an important role in protecting gastric mucosa from aggressive agents [55]. Various ulcerogenic agents have been reported to induce tissue damage by decreasing the endogenous NP-SH level [56]. It is known that ethanol exerts its aggressive effect on the gastric mucosa by diminishing endogenous NP-SH content [57]. NP-SH participates in controlling the production and nature of the mucus in order to protect the gastric mucosa from the noxious effect of ROS formation due to ethanol administration [58]. Our study shows that the DES pre-treatment significantly inhibited ethanol-induced NP-SH depletion when compared to the ulcer control group. Therefore, it could be proposed that replenishment of the endogenous NP-SH might contribute in the gastroprotective activity of DES.

The article "Gastroprotective effect of desmosdumotin C isolated from Mitrella kentii against ethanol-induced gastric mucosal hemorrhage in rats: possible involvement of glutathione, heat-shock protein-70, sulfhydryl compounds, nitric oxide, and anti-Helicobacter pylori activity" was retracted in 2024. Reasons: duplicated images; overlap with earlier publications; unreliable results or conclusions; concerns about the authorship.

Prostaglandins (PGs) play an important role in the maintenance of mucosal integrity which is formed by the COX isoenzymes, namely COX-1 and COX-2 isoforms. Recent studies have found that PGs biosynthesis in the gastrointestinal tract is exclusively catalyzed by COX-1, whereas COX-2 mainly yields PGs in pathophysiological reactions such as inflammation [59]. Independent of PGs, other protective factors involved in the maintenance of mucosal integrity include NO and heat shock proteins [60]. Under normal conditions, NO is formed by nitric oxide synthase (NOS). Neuronal NOS (nNOS) constitutively produces NO, whereas inducible NOS (iNOS) forms NO under inflammatory gastrointestinal damage [61]. On the other hand, activation of HSP-70 suppresses gastric iNO synthesis [45]. The relation between COX-2 and NO at the inflammatory condition was well documented [62] and experimentally in animal models, mucosal injury was found to be accompanied with COX-2 expression [63] as well as inducible nitric oxide (iNO) [64]. Accordingly, the control of stomach ulceration was observed to be achieved by the suppression of inflammatory mediators [65]. It is important to mention that selective COX-2 inhibitors do not damage normal gastric mucosa. However, severe gastric damage occurs when COX-2 inhibition is accompanied by suppression of NO formation or defunctionalization of the afferent nerves [59]. Thus, to evaluate the cytoprotective activity of DES, its effect on COX-2/NO system was evaluated. DES interfered with COX-2 inflammatory pathway and NO level. It is interesting to discover a compound with combined anti-inflammatory and anti-ulcer activities, taking into account the serious limitations of many anti-inflammatory agents that show deleterious effects on the stomach, resulting in gastric mucosal damage [66].

The article "Gastroprotective effect of desmosdumotin C isolated from Mitrella kentii against ethanol-induced gastric mucosal hemorrhage in rats: possible involvement of glutathione, heat-shock protein-70, sulfhydryl compounds, nitric oxide, and anti-Helicobacter pylori activity" was retracted in 2024. Reasons: duplicated images; overlap with earlier publications; unreliable results or conclusions; concerns about the authorship.

The microaerophilic bacterium *H pylori* is a gram negative bacilliform considered to be one of the main etiologic factors in the development of the peptic ulcer disease [67]. The bacterium infection results from its induction effect on inflammatory cells to the gastric mucosa [68], without invading the gastric epithelium [69]. Currently, common anti *H pylori* regimen therapies pose side effects. Therefore, the need to discover new agents with potential anti *H pylori* activity is of high concern [70]. A potent antibacterial compound is one that shows an MIC value of less than or equal to 250 [71]. To evaluate the antimicrobial activity of DES, the compound was examined against *H pylori* strains and the result of the present study showed an interesting DES MIC value of 125 μg/ml against *H. pylori* J99.

## Conclusions

The current study introduces, for the first time, the isolation of DES compound from *M. kentii* plant and the evaluation of its gastroprotective activity against ethanol-induced gastric ulcer. The possible gastroprotective mechanism(s) of DES might be attributed to the intracellular antioxidant effect revealed by lowered MDA levels and restored GSH levels, besides HSP-70 up regulation. Moreover, DES exhibited anti-apoptotic activity marked by the down regulation of Bax protein. Furthermore, DES was found to maintain endogenous NP-SH content. The compound inhibited COX-2 activity and replenished the NO level. It also showed an interesting MIC against *H Pylori* bacterium. These results warrant further study on DES compound as an effective gastroprotective and therapeutic agent for gastric ulcer.

## Abbreviations

M.kentii: Mitrella kentii; DES: Desmosdumotin C; TXB 2: Thromboxane B 2; PAF: Platelet activating factor; NP-SH: Non protein sulfhydryl; COX-2: Cycloxygenase-2 enzyme; NO: Nitric oxide; MDA: Malondialdehyde; GSH: Glutathione; HSP: Heat shock protein; Bcl2: B-cell lymphoma 2; Bax: Bcl-2–associated X protein; HE: Hematoxylene and eosin; PAS: Periodic acid schiff base; IHC: Immunhistochemistry; H pylori: Helicobacter pylori; AST: Aspartate transaminase; ALT: Alanine aminotranferase; DTNB: 5,5 -dithiobis-2-nitrobenzoic acid; TBARS: Thiobarbituric acid reactive substance; FRAP: Ferric-reducing antioxidant power; S.E.M: Standard error mean; ANOVA: Analysis of variance; MIC: Minimum inhibitory concentration; PBS: Phosphate buffered saline.

## Competing interests

The authors declare that they have no competing interests.

The article "Gastroprotective effect of desmosdumotin C isolated from Mitrella kentii against ethanol-induced gastric mucosal hemorrhage in rats: possible involvement of glutathione, heat-shock protein-70, sulfhydryl compounds, nitric oxide, and anti-Helicobacter pylori activity" was retracted in 2024. Reasons: duplicated images; overlap with earlier publications; unreliable results or conclusions; concerns about the authorship.

## Authors’ contributions

HMS drafted the manuscript and performed the toxicity study, gastroprotective study, COX-2 activity study and gastric homogenate contents estimation. AA, AAH and KAK carried out the extraction and isolation of the compound. SM performed the statistical analysis and revised the manuscript critically for important intellectual content. MAA, SIA, NMH participated in the design of the study. MMT performed the Immunhistochemistry staining. MFL and JV carried out the *H pylori* study. All authors read and approved the final manuscript.

## Pre-publication history

The pre-publication history for this paper can be accessed here:

http://www.biomedcentral.com/1472-6882/13/183/prepub
